The article "Bioinformatics Analysis of ceRNA Network Related to Polycystic Ovarian Syndrome" was published in 2021. Journal: Comput Math Methods Med.

# Bioinformatics Analysis of ceRNA Network Related to Polycystic Ovarian Syndrome

**DOI:** 10.1155/2021/9988347

**Published:** 2021-06-09

**Authors:** Yuanqi Li, Yong Tan

**Affiliations:** ^1^Nanjing University of Chinese Medicine, Nanjing, Jiangsu 210029, China; ^2^Affiliated Hospital of Nanjing University of Chinese Medicine, Nanjing, Jiangsu 210029, China

## Abstract

**Introduction:**

Polycystic ovary syndrome (PCOS) is caused by the hormonal environment in utero, abnormal metabolism, and genetics, and it is common in women of childbearing age. A large number of studies have reported that lncRNA is important to the biological process of cancer and can be used as a potential prognostic biomarker. Thus, we studied lncRNAs' roles in PCOS in this article.

**Methods:**

We obtained mRNAs', miRNAs', and lncRNAs' expression profiles in PCOS specimens and normal specimens from the National Biotechnology Information Gene Expression Comprehensive Center database. The EdgeR software package is used to distinguish the differentially expressed lncRNAs, miRNAs, and mRNAs. Functional enrichment analysis was carried out by the clusterProfiler R Package, and the lncRNA-miRNA-mRNA interaction ceRNA network was built in Cytoscape plug-in BiNGO and Database for Annotation, Visualization, and Integration Discovery (DAVID), respectively.

**Results:**

We distinguished differentially expressed RNAs, including 1087 lncRNAs, 14 miRNAs, and 566 mRNAs in PCOS. Among them, 410 lncRNAs, 11 miRNAs, and 185 mRNAs were contained in the ceRNA regulatory network. The outcomes from Gene Ontology (GO) analysis showed that the differentially expressed mRNAs (DEMs) were mainly enriched in response to the maternal process involved in female pregnancy, morphogenesis of embryonic epithelium, and the intracellular steroid hormone receptor signaling pathway. The Kyoto Encyclopedia of Genes and Genomes (KEGG) pathway analysis data showed that DEMs were primarily enriched in pathways related to the TGF-*β* signaling pathway, Type I diabetes mellitus, and glycolysis/gluconeogenesis. In addition, we chose NONHSAT123397, ENST00000564619, and NONHSAT077997 as key lncRNAs due to their high bearing on PCOS.

**Conclusion:**

ceRNA networks play an important role in PCOS. The research indicated that specific lncRNAs were related to PCOS development. NONHSAT123397, ENST00000564619, and NONHSAT077997 could be regarded as potential diagnostic mechanisms and biomarkers for PCOS. This discovery might provide more effective and more novel insights into the mechanisms of PCOS worthy of further exploration.

## 1. Introduction

Polycystic ovary syndrome (PCOS) is caused by the hormonal environment in utero, abnormal metabolism, and genetics, and its incidence is related to race and eating habits [1–3]. The disease is very common in women of childbearing age, and its common clinical symptoms include menstrual disorders, hirsutism, obesity, and infertility [4–10]. Among them, according to relevant statistics, obesity accounts for 30% to 60% of PCOS patients. PCOS is often accompanied by other diseases, such as diabetes, cardiovascular disease (CVDS), and other complications [11–13]. The current treatment methods are mainly oral contraceptives and drugs to reduce hyperandrogenemia [14], ovulation-stimulating drugs [15, 16], surgical treatment, and *in vitro* fertilization [17]. Since the cause of the disease is not yet clear, the clinical treatment of PCOS patients also has limitations. Therefore, more research on the pathogenesis of PCOS is needed to find efficient biomarkers.

The article "Bioinformatics Analysis of ceRNA Network Related to Polycystic Ovarian Syndrome" was published in 2021. Journal: Comput Math Methods Med.

Long noncoding RNAs (lncRNAs) are noncoding RNAs longer than 200 nucleotides [18, 19]. A large number of researches have shown that lncRNA is important to the biological process of cancer and can be used as a potential prognostic biomarker. The different mechanisms of lncRNA action in cancer will lead to different expression patterns in cancer cells. For example, according to related reports by Li et al., lncRNA GAS5 was upregulated in PCOS and could participate in the occurrence of diseases by regulating cell apoptosis and IL-6 expression [20]. Qin et al. proved for the first time that lncRNA H19 was associated with PCOS, which was a useful biomarker for early endocrine and metabolic abnormalities in PCOS [21]. Liu et al. found that the expression of lncRNA-Xist was related to the pathogenesis of PCOS. Knocking down the expression of this gene in PCOS could lead to the proliferation and migration of cancer cells [22]. Further secrets about lncRNA in cancers remain to be discovered.

There is increasing evidence that noncoding RNA (ncRNA) plays a key role in the development of human diseases [23]. Many studies have shown that these ncRNAs participate in competitive regulatory interactions [24]; that is, a network of competitive endogenous RNAs (ceRNAs) and lncRNAs can act as microRNA bait to regulate gene expression [25]. These interactions are usually interconnected, so any abnormal expression of network components may derail complex regulatory circuits and ultimately lead to the development and progression of cancer. According to reports, XLOC_006390 acts as a ceRNA and reversely regulates the expression of miR-331-3p and miR-338-3p, thereby promoting the occurrence and metastasis of cervical cancer [26]. MT1JP regulates the progression of gastric cancer by acting as a ceRNA to competitively bind to miR-92a-3p and regulate the expression of FBXW7 [27].

The article "Bioinformatics Analysis of ceRNA Network Related to Polycystic Ovarian Syndrome" was published in 2021. Journal: Comput Math Methods Med.

Herein, just as Figure 1 shows, we build a global triple network through the National Center for Biotechnology Information and Gene Expression Omnibus (NCBI and GEO) data. Research design is based on the internal competitive endogenous RNA (ceRNA) theory, and bioinformatics analysis is conducted to explore PCOS in the lncRNA-miRNA-mRNA network.

## 2. Materials and Methods

### 2.1. PCOS Data

GEO (https://www.ncbi.nlm.nih.gov/geo/query/acc.cgi), an open-access functional genomics database, offers support for the submission of MIAME-compatible data. GEO could provide data based on arrays and sequences as well as tools to help users download gene expression profiles. We downloaded the human miRNA real-time PCR array database in GEO (GSE37425).

### 2.2. lncRNAs', miRNAs', and mRNAs' Differentially Expressed Screening

The differentially expressed lncRNAs (DELs), miRNAs (DEMis), and mRNAs (DEMs) between normal tissue and PCOS tissue are set out through a two-level differential method. Then, the differentially expressed genes were screened by *t*-test. In light of *P* values less than 0.05 and fold change more than 2, we screened the data from DELs, DEMis, and DEMs.

### 2.3. lncRNAs and mRNAs of DEMis Determination

RNAhybrid and miRanda were employed to determine lncRNAs' miRNA targets and measure free energy (MFE) of miRNA-lncRNA double-stranded bodies' minimum value. We found miRNA sequences in miRBase (http://www.mirbase.org/) and checked lncRNA sequences in NCBI (https://www.ncbi.nlm.nih.gov/) nucleotides. miRNA target binding sites were determined across the total lncRNA sequence. We chose lncRNAs with perfect nucleotides to pair at the 2nd and 8th ends of miRNA sequences to gain high-quality lncRNAs, and we then selected these lncRNAs to act as miRNA targets. We downloaded data about miRNA-mRNA interactions from miRTarBase (http://mirtarbase.cuhk.edu.cn/php/index.php) and miRWalk (http://mirwalk.umm.uni-heidelberg.de/).

### 2.4. Building of the lncRNA-miRNA-mRNA Network

On the basis of the ceRNA theory to build the lncRNA-miRNA-mRNA network, the methods were as follows: (1) We selected Pearson's correlation coefficient (PCC) to determine the correlation between the DELs' and DEMs' expression. The coexpressed lncRNA-mRNA pairs' standard was PCC more than 0.99 and *P* less than 0.05. (2) The coexpression of a competition triplet was identified when mRNA and lncRNA in a pair were both targeted to a certain common miRNA and negatively expressed. (3) Next, coexpression competing triads were assembled to reconstruct the lncRNA-miRNA-mRNA network using Cytoscape software for visualization. Meanwhile, the degrees of all nodes in the miRNA-lncRNA-mRNA network were determined.

The article "Bioinformatics Analysis of ceRNA Network Related to Polycystic Ovarian Syndrome" was published in 2021. Journal: Comput Math Methods Med.

### 2.5. Analysis of Functional Enrichment

In functional enrichment analysis, the Cytoscape plug-in BiNGO and Database for Annotation, Visualization, and Integration Discovery Database (DAVID, https://david.ncifcrf.gov/) were used to perform Gene Ontology (GO) biological process terminology and Kyoto Encyclopedia of Genes and Genomes (KEGG) pathway analyses on mRNAs in the lncRNA-miRNA-mRNA network, respectively. Then, we used Cytoscape plug-in BiNGO to rebuild the GO interactive network.

### 2.6. Key lncRNA-miRNA-mRNA Subnetwork Rebuilding

We extracted each lncRNA of the global triple network and its connected miRNAs and mRNAs, which were prepared for Cytoscape software to rebuild the new subnetwork. At the same time, the lncRNA-miRNA first and second relationship pairs' number was calculated. Next, we collected key lncRNAs by lncRNA node number, first and second relationship pairs' number, and lncRNA-miRNA's quantity. Further, every last key lncRNA was used to perform GO and pathway annotations. Then, Cytoscape plug-in BiNGO was selected to reconstruct the GO interactive network.

## 3. Results

### 3.1. Data Preprocessing

The human miRNA real-time PCR array database included 14 miRNAs, and 10 coexpression miRNAs were selected in this study. There were 566 mRNAs and 1087 lncRNAs selected in the human lncRNA/mRNA microarray data.

### 3.2. Results of DELs', DEMs', and DEMis' Screening

We chose to preprocess data by *P* values less than 0.05 and fold change more than 2. 566 differentially expressed mRNAs (DEMs), 1087 differentially expressed lncRNAs (DELs), and 14 differentially expressed miRNAs (DEMis) were filtered. Next, we merged the DEMs and DELs with the target mRNAs and lncRNAs of DEMis, respectively. We got 410 coexpression lncRNAs, 185 coexpression mRNAs, and 10 DEMis. Lastly, we chose these genes for reconstructing the lncRNA-miRNA-mRNA network.

### 3.3. lncRNA-miRNA-mRNA Network

For evaluating the lncRNAs' features as targets of miRNA, we first reconstructed and then visualized the network between lncRNAs and miRNAs. As shown in Figure 2, there were 410 lncRNAs, 11 miRNAs, and 691 edges in the network. Then, we also reconstructed the network between miRNAs and mRNA. As shown in Figure 3, there were 10 miRNAs, 185 mRNAs, and 449 edges in this network. Finally, we rebuilt the lncRNAs', miRNAs', and mRNAs' networks. As shown in Figure 4, there were 410 lncRNAs, 185 mRNAs, 10 miRNAs, and 1079 edges in the lncRNA-miRNA-mRNA network.

### 3.4. Prediction of lncRNA Function Based on lncRNA-miRNA-mRNA Network

We observed that one or more mRNAs surround and bind to lncRNAs in the lncRNA-miRNA-mRNA network. Thus, we could infer each lncRNA function according to the connected mRNAs' features. We analyzed the DEL functions by all DEMs. For a deeper understanding of the function of DEMs in PCOS, we used the BiNGO plug-in to enrich the functions of these DEMs. The results of GO analysis revealed that the DEMs were enriched in 526 biological process (BP) terms, particularly in sodium ion transport, response to interferon-gamma, neural tube development, morphogenesis of embryonic epithelium, leukocyte chemotaxis, antigen processing, presentation of peptide, and more. The DEMs were enriched in 104 molecular function (MF) terms, such as virus receptor activity, Ras guanyl-nucleotide exchange factor activity, and guanyl-nucleotide exchange factor activity. The DEMs were enriched in 91 cellular component (CC) terms, such as filopodium, lamellipodium, and axon terminus. The top thirty significant GO terms are listed in Figure 5 according to *P* value. Additionally, KEGG pathway analysis indicated that 97 pathways especially related to TGF-*β* signaling, Type I diabetes mellitus, and glycolysis/gluconeogenesis were obviously enriched. The top thirty significant KEGG pathways are shown in Figure 6 according to *P* value.

The article "Bioinformatics Analysis of ceRNA Network Related to Polycystic Ovarian Syndrome" was published in 2021. Journal: Comput Math Methods Med.

### 3.5. Topological Analysis of the PCOS-Related lncRNA-miRNA-mRNA Network

Hub nodes are important to biological networks. Thus, we explored all nodes' degrees in the lncRNA-miRNA-mRNA network. Based on the previous research from Hanet al., a node degree exceeding 5 was defined as a hub node. As shown in Table 1 and Figure 7, 30 nodes containing 10 lncRNAs, 10 miRNAs, and 10 mRNAs could be selected as hub nodes in this study. Moreover, the quantity of the lncRNA-miRNA pairs and the miRNA-mRNA pairs are counted and shown in Table 2. We observed NONHSAT123397, ENST00000564619, and NONHSAT077997. We found that they had higher degrees of nodes and a higher quantity of pairs. These results suggested that they played a key role in the launch and progress of PCOS; thus, they were selected as the key lncRNAs.

### 3.6. Subnetwork of Key lncRNA-miRNA-mRNA

As we all know, lncRNAs and mRNAs have a common coexpression mode in the ceRNA network. Therefore, we picked up the key lncRNAs and their linked mRNAs and miRNAs from the previous lncRNA-miRNA-mRNA network and reconstructed the subnetworks of key lncRNAs-miRNAs-mRNAs. As presented in Figures 8–10, the lncRNA NONHSAT123397-miRNA-mRNA subnetwork covered 7 miRNA nodes, 143 mRNAs, and 358 edges; the lncRNA ENST00000564619-miRNA-mRNA subnetwork covered 6 miRNAs, 140 mRNAs, and 304 edges; and the lncRNA NONHSAT077997-miRNA-mRNA subnetwork covered 6 miRNAs, 139 mRNAs, and 320 edges. Analysis of the GO terms and KEGG pathways demonstrated that 550 GO terms and 80 pathways were enriched in the subnetwork of NONHSAT123397, 553 GO terms and 82 pathways were enriched in the subnetwork of ENST00000564619, and 533 GO terms and 80 pathways were enriched in the subnetwork of NONHSAT077997. The top 30 significantly enriched GO terms and KEGG pathways of each subnetwork are listed in Figures 11–13.

The article "Bioinformatics Analysis of ceRNA Network Related to Polycystic Ovarian Syndrome" was published in 2021. Journal: Comput Math Methods Med.

## 4. Discussion

PCOS has become a common disease in women, and the metabolic abnormalities of many PCOS patients often lead to the risk of cardiovascular disease [28, 29]. In recent years, there have been many controversies about the oncogene of PCOS. Many studies have shown that insulin deficiency may be the main cause of PCOS [30, 31]. In addition, obesity is also considered the main cause. More than 30% of PCOS patients suffer from obesity, and obesity makes the clinical treatment of PCOS more difficult. However, the exact reason for PCOS is still unclear. Currently, therapies like oral contraceptives can regulate menstruation and reduce the production of adrenal androgens [32, 33], but they can only be used for women who have no plan to be pregnant. In short, more research and therapies targeting the pathogenesis and pathophysiology of PCOS need to be explored.

Different from coding RNAs, lncRNAs' functions have not been well studied, and the exploration of lncRNAs' functions is full of challenges. Recently, accumulated data have found that lncRNAs had abnormal expressions in many diseases [34], such as PCOS, which indicates that lncRNA might have a special role in disease progression. So far, some studies have found that lncRNAs exert their functions by regulating mRNA expression or binding with miRNAs. For example, Luo et al. found lncRNA CASC11 might increase the capability of bladder cancer cell proliferation, and the roles of lncRNA CASC11 are probably through miRNA-150 [35]. Wang et al. showed that lnc00152 slicing repressed the growth and invasiveness of hemangioma cells by regulating miR-139-5p [36]. Besides, some studies point out that the relation among lncRNA, miRNA, and mRNA is worth exploring in cancer development [37, 38]. Similarly, Wu et al. discussed the therapeutic extent and role of miRNA, lncRNA, and circRNA in osteoarthritis [39].

The ceRNA (competing endogenous RNA) hypothesis prompts a novel mechanism of RNAs' interaction [40]. miRNA can silence genes through binding to mRNA [41], and ceRNA can adjust gene expression through binding to miRNA competitively [42]. Compared with the miRNA regulatory network, the ceRNA regulatory network is more sophisticated and complex, involving more RNA molecules, including mRNA, pseudogenes of coding genes, long noncoding RNAs, and miRNAs [43]. It provides a new perspective for scientific researchers to conduct transcriptome research. Thus, the purpose of this research is to determine the function and inner mechanism of lncRNAs as ceRNAs in PCOS through the lncRNA-miRNA-mRNA network.

The article "Bioinformatics Analysis of ceRNA Network Related to Polycystic Ovarian Syndrome" was published in 2021. Journal: Comput Math Methods Med.

Herein, we downloaded PCOS data in the NCBI GEO database. Based on a theory about ceRNA that the lncRNAs and mRNAs share the same miRNAs in triplets, we then established a global triple network by these data about PCOS. We determined 1087 lncRNAs, 14 miRNAs, and 566 mRNAs as differentially expressed RNAs. Meanwhile, we discovered that the lncRNA-miRNA-mRNA network was composed of 410 lncRNAs, 11 miRNAs, and 185 mRNAs. We evaluated the biological functions enriched in differentially expressed coding genes through Gene Ontology (GO) analysis and pathway analysis. We chose GO analysis as a control track for exploring the differentially expressed genes' function and depicted the distribution of genes and gene products. According to the precise test of KEGG and Fisher's and the significance threshold defined by the *P* value, pathway analysis was applied to the differentially expressed genes' location. The GO analysis' results showed that the differentially expressed mRNAs (DEMs) were mainly rich in the following aspects: response to the maternal process involved in female pregnancy, morphogenesis of embryonic epithelium, and the intracellular steroid hormone receptor signaling pathway. The Kyoto Encyclopedia of Genes and Genomes (KEGG) pathway analysis results indicated that DEMs were mostly enriched in the TGF-*β* signaling pathway, Type I diabetes mellitus, and glycolysis/gluconeogenesis.

These important GO clauses involved in the maternal course were involved in response to interferon-gamma [44], neural tube development [45], morphogenesis of embryonic epithelium, leukocyte chemotaxis, antigen processing, presentation of peptide, and more [46–48]. The pathway analysis indicated that 97 pathways got rich, and it mainly involved the TGF-*β* signaling pathway [49, 50], Type I diabetes mellitus [51], and glycolysis/gluconeogenesis [52, 53]. All pathways determined were important to PCOS. Research on lncRNAs is getting much deeper, due to the expression of lncRNA related to its functions. Thus, lncRNAs are more suitable as reliable and effective biomarkers and therapeutic targets. Lately, many researchers have found several lncRNA-focused features to increase the cure rate of certain diseases, but lncRNAs' diagnostic role in PCOS has not been fully studied. We used the hub nodes and the relationship pairs' quantity to find key lncRNAs as new potential biomarkers for PCOS diagnosis and prognosis. Some studies have shown that hub nodes, which are characterized by their high connectivity with others, can be regarded as the network for accessing genes of importance [54]. Generally, lncRNAs with more relationship pairs show that lncRNAs are hubs involved in ceRNA interplay [55, 56]. Therefore, lncRNA is indispensable and important for network organization.

The article "Bioinformatics Analysis of ceRNA Network Related to Polycystic Ovarian Syndrome" was published in 2021. Journal: Comput Math Methods Med.

It has been observed that NONHSAT123397, ENST00000564619, and NONHSAT077997 are the key nodes of the topology. The amount of lncRNA-miRNA and miRNA-mRNA pairs and the number of nodes far exceed other lncRNAs. These lncRNAs are important to PCOS and can be regarded as key lncRNAs. In the midst of these key lncRNAs, NONHSAT123397 is a rarely reported lncRNA. It has many functions, including connecting many mRNAs and interacting with many miRNAs known to be involved with PCOS. NONHSAT123397 is also related to PCOS due to the results of GO and pathway analyses, so these indicate that NONHSAT123397 is a key lncRNA to PCOS. However, the function of NONHSAT123397 to PCOS is not currently indicated from the current studies. On the basis of the subnetwork of NONHSAT123397-miRNA-mRNA, we speculate that NONHSAT123397 might compete with certain miRNA families to cause changes in the expression of downstream mRNAs linked to PCOS, like the miR-3135b and miR-3188 families. In order to confirm our guess, experiments in recent years have shown that miR-3135b and miR-3188 families are critical for PCOS's development [57]. For example, Wang et al. indicated that miR-3188 and miR-3135b in granulosa cells of PCOS patients were negatively correlated with FSH, while miR-3188 was positively correlated with BMI, and hsa-miR-3188/3135b improved the prediction accuracy of PCOS [58]. In addition, studies show that the TGF-*β* signaling pathway is important to PCOS. Meanwhile, the target genes corresponding to miRNA-3135b are highly enriched in the TGF-*β* signaling pathway and insulin secretion. Downregulation of miR-486-5p expression in cumulus cells of metaphase II oocytes in patients with the polycystic ovary syndrome could control the proliferation of cumulus cells by activating PI3K/Akt.

This study has some limitations. The current experimental data are not enough to enable us to have a comprehensive understanding of the mechanism of action of these three lncRNAs, so we need to continue to explore. In future studies, we will collect more clinical samples, and we will explore the correlation between the expression of NONHSAT123397, ENST00000564619, and NONHSAT077997 and clinical parameters (including age, clinical stage, and survival time). Secondly, we will explore the regulation of the proliferation and metastasis of PCOS by NONHSAT123397, ENST00000564619, and NONHSAT077997. Finally, the ceRNA network identified in this study will be verified through experiments, such as through the dual-luciferase assay and the RNA immunoprecipitation assay.

The article "Bioinformatics Analysis of ceRNA Network Related to Polycystic Ovarian Syndrome" was published in 2021. Journal: Comput Math Methods Med.

## 5. Conclusion

Studies have shown that the development trend of PCOS in the human body will be affected by specific lncRNAs. Our research revealed that the ceRNA network, which involves a new type of interaction between lncRNAs, miRNAs, and mRNAs, have the potential to influence the occurrence and development of PCOS disease. The significant differential expression of NONHSAT123397, ENST00000564619, and NONHSAT077997 in PCOS means that these three genes may play an important role in PCOS. Then, we have a further breakthrough in the mechanism of PCOS. In short, in this experiment, we have discovered a new therapeutic target for PCOS, which is a new breakthrough in the treatment of clinical PCOS patients.

## Figures and Tables

**Figure 1:** The reconstruction of the lncRNA-miRNA-mRNA network. Firstly, expression data of miRNA, lncRNA, and mRNA were downloaded from the Gene Expression Omnibus. Secondly, DEMs (differentially expressed mRNAs), DELs (differentially expressed lncRNAs), and DEMis (differentially expressed miRNAs) were screened at ∣fold change)∣>2 and false discovery rate (FDR) < 0.05. Thirdly, target lncRNAs of DEMis were predicted using RNAhybrid and miRanda, and target mRNAs of DEMis were predicted using miRTarBase and miRWalk. Fourthly, the coexpression lncRNAs and coexpression mRNAs were obtained to merge the target lncRNAs and mRNAs of DEMis with DELs and DEMs, respectively. Finally, the coexpression lncRNAs, DEMis, and coexpression mRNAs were mapped into the interactions.

**Figure 2:** The lncRNA-miRNA interaction network. There were 410 lncRNAs, 11 miRNAs, and 691 edges in the network. The square stands for lncRNA and the circle stands for miRNA. All shapes in red stand for upregulation, and green stand for downregulation.

**Figure 3:** The miRNA-mRNA interaction network. There were 10 miRNAs, 185 mRNAs, and 449 edges in the network. The rhombus stands for mRNA, and the circle stands for miRNA. All shapes in red stand for upregulation, and those in green stand for downregulation.

**Figure 4:** The dysregulated lncRNA-mRNA-miRNA ceRNA network. There were 410 lncRNAs, 10 miRNAs, 185 mRNAs, and 1079 edges in the network. The square stands for lncRNA, the rhombus stands for mRNA, and the circle stands for miRNA. All shapes in red stand for upregulation, and those in green stand for downregulation.

**Figure 5:** The enriched GO terms of the genes involved in the ceRNA network in PCOS. The *x*-axis stands for the enrichment factor of the indicated genes, and the *y*-axis stands for the top 30 GO terms. The circle denotes the biological process term, the triangle denotes the cellular component term, and the square denotes the molecular function term. The gradient of green to red denotes a change in the significance of the correlation from low to high. The different sizes of the dots denote related mRNA numbers.

The article "Bioinformatics Analysis of ceRNA Network Related to Polycystic Ovarian Syndrome" was published in 2021. Journal: Comput Math Methods Med.

**Figure 6:** The enriched KEGG pathways of the genes involved in the ceRNA network in PCOS. The *x*-axis stands for the enrichment factor of the indicated genes, and the *y*-axis stands for the top 30 KEGG pathways. The circle denotes the biological process term, the triangle denotes the cellular component term, and the square denotes the molecular function term. The gradient of green to red denotes a change in the significance of the correlation from low to high. The different sizes of the dots denote related mRNA numbers.

**Figure 7:** All node degree analysis reveals specific properties of the lncRNA-miRNA-mRNA network.

**Figure 8:** The subnetwork of lncRNA NONHSAT123397. The square stands for lncRNA, the rhombus stands for mRNA, and the circle stands for miRNA. All shapes in red stand for upregulation, and those in green stand for downregulation.

**Figure 9:** The subnetwork of lncRNA ENST00000564619. The square stands for lncRNA, the rhombus stands for mRNA, and the circle stands for miRNA. All shapes in red stand for upregulation, and those in green stand for downregulation.

**Figure 10:** The subnetwork of lncRNA NONHSAT077997. The square stands for lncRNA, the rhombus stands for mRNA, and the circle stands for miRNA. All shapes in red stand for upregulation, and those in green stand for downregulation.

**Figure 11:** The top 30 significantly enriched GO terms (a) and KEGG pathways (b) of lncRNA NONHSAT123397-miRNA-mRNA subnetwork-related mRNAs.

**Figure 12:** The top 30 significantly enriched GO terms (a) and KEGG pathways (b) of lncRNA ENST00000564619-miRNA-mRNA subnetwork-related mRNAs.

**Figure 13:** The top 30 significantly enriched GO terms (a) and KEGG pathways (b) of lncRNA NONHSAT077997-miRNA-mRNA subnetwork-related mRNAs.

**Table 1:** The list of differentially expressed genes (node degree 45).

Number	Gene name	Node degree	Gene type	Fold change
1	Hsa-miR-3135b	248	mi	1.180132215
2	Hsa-miR-4758-5p	163	mi	1.121940431
3	Hsa-miR-4749-5p	131	mi	1.045117605
4	Hsa-miR-4649-5p	121	mi	1.124608718
5	Hsa-miR-3188	110	mi	1.475727733
6	Hsa-miR-1231	105	mi	1.205829903
7	Hsa-miR-455-3p	66	mi	1.000930169
8	Hsa-miR-486-5p	66	mi	1.051809938
9	Hsa-miR-4286	37	mi	-1.037989108
10	Hsa-miR-3609	32	mi	1.043174805
11	PAFAH1B2	8	m	-1.1099555
12	CFLAR	8	m	-1.076701125
13	NONHSAT123397	7	lnc	-2.415788663
14	MSR1	7	m	-2.200573263
15	ABL2	7	m	-1.399022013
16	TPM3	7	m	-1.386117525
17	FKBP5	7	m	-1.33889315
18	PEX5L	6	m	-1.940342225
19	AAK1	6	m	-1.661734963
20	RAB3IP	6	m	-1.554929325
21	ENST00000564619	6	lnc	-1.464096138
22	NONHSAT077997	6	lnc	-1.316733238
23	AKAP5	6	m	-1.24698225
24	NONHSAT145473	5	lnc	-1.4293997
25	NONHSAT104609	5	lnc	-1.2225913
26	NR_027512.1	5	lnc	-1.21770025
27	FR233072	5	lnc	-1.104499363
28	NONHSAT083947	5	lnc	-1.08422
29	NONHSAT026319	5	lnc	-1.052942563
30	NONHSAT033305	5	lnc	-2.450632488

The article "Bioinformatics Analysis of ceRNA Network Related to Polycystic Ovarian Syndrome" was published in 2021. Journal: Comput Math Methods Med.

**Table 2:** The number of lncRNA-miRNA and miRNA-mRNA pairs.

Gene name	lncRNA-miRNA pairs	miRNA-mRNA pairs	Total number
NONHSAT123397	7	313	320
ENST00000564619	6	298	304
NONHSAT077997	6	352	358
NONHSAT145473	5	252	257
NONHSAT104609	5	252	257
NR_027512.1	5	252	257
FR233072	5	263	268
NONHSAT083947	5	257	262
NONHSAT026319	5	251	256
NONHSAT033305	4	179	183

## Data Availability

The data that support the findings of this study are available with approval from the authors.
